The article "Inhibitory Effect of Long-Chain Fatty Acids on Biogas Production and the Protective Effect of Membrane Bioreactor" was published in 2016. Journal: Biomed Res Int.

# Inhibitory Effect of Long-Chain Fatty Acids on Biogas Production and the Protective Effect of Membrane Bioreactor 

**DOI:** 10.1155/2016/7263974

**Published:** 2016-09-08

**Authors:** Kris Triwulan Dasa, Supansa Y. Westman, Ria Millati, Muhammad Nur Cahyanto, Mohammad J. Taherzadeh, Claes Niklasson

**Affiliations:** ^1^Department of Food and Agricultural Product Technology, Universitas Gadjah Mada, Yogyakarta 55281, Indonesia; ^2^Swedish Center for Resource Recovery, University of Borås, 50190 Borås, Sweden; ^3^Department of Chemistry and Chemical Engineering, Chalmers University of Technology, 41296 Gothenburg, Sweden

## Abstract

Anaerobic digestion of lipid-containing wastes for biogas production is often hampered by the inhibitory effect of long-chain fatty acids (LCFAs). In this study, the inhibitory effects of LCFAs (palmitic, stearic, and oleic acid) on biogas production as well as the protective effect of a membrane bioreactor (MBR) against LCFAs were examined in thermophilic batch digesters. The results showed that palmitic and oleic acid with concentrations of 3.0 and 4.5 g/L resulted in >50% inhibition on the biogas production, while stearic acid had an even stronger inhibitory effect. The encased cells in the MBR system were able to perform better in the presence of LCFAs. This system exhibited a significantly lower percentage of inhibition than the free cell system, not reaching over 50% at any LCFA concentration tested.

## 1. Introduction

Comprising mainly methane, biogas is a renewable energy source that can be directly used as a car fuel, for heating, or indirectly used to generate electricity [1]. Biogas production through anaerobic digestion involves four crucial steps including hydrolysis, acidogenesis, acetogenesis, and methanogenesis. Each step is carried out by different consortia of microorganisms, partly standing in syntrophic interrelation with each other [2]. Biogas can be produced from various kinds of waste materials, including municipal solid waste (MSW), industrial waste, and agricultural waste. Among waste materials, lipid-rich wastes, which are released from, for example, dairy products industry, slaughterhouses, edible oil processing industry, olive oil mills, and wool scouring facilities are produced in high amounts each year [3–6]. Accumulation of this waste creates a serious problem to the environment such as heavy odor and plenty of leachate; hence, a sustainable handling of this waste is highly desirable.

Lipids, the main constituent in lipid-rich wastes, play the most significant role in anaerobic digestion for biogas production due to their high energy content [7]. Lipids are long-chain fatty acids (LCFAs) bonded to glycerol, alcohols, or other groups by an ester or ether linkage. During hydrolysis, lipids are rapidly degraded into monomers such as glycerol and LCFAs which are further converted into short organic acids via *β*-oxidation [7]. The short organic acids are subsequently converted into acetate and hydrogen which are eventually converted into methane and carbon dioxide [1]. Biogas derived from lipid have higher methane content compared to that derived from carbohydrates and proteins [7].

The article "Inhibitory Effect of Long-Chain Fatty Acids on Biogas Production and the Protective Effect of Membrane Bioreactor" was published in 2016. Journal: Biomed Res Int.

Albeit the higher quality of biogas produced from lipid, biogas production from lipid is hampered by excessive organic loading or LCFAs [8, 9]. It has been reported that LCFAs inhibited several reactions during the anaerobic degradation process [10]. The inhibitory effects of LCFA are already visible at concentrations as low as 50 mg/L [11]. LCFAs also have severe inhibitory effects on the microorganisms in anaerobic digestion, particularly for methanogens and acetogens [11].

Another challenge in the anaerobic digestion process of lipid-containing wastes is washout of methanogens at high organic loading rates. Methanogens grow very slow and sensitive in the harsh process conditions. As a result, methanogens require longer retention time in the digesters [12]. In addition, methanogens is also sensitive to inhibitor compound. Sousa et al. [13] reported that methanogens in the anaerobic digestion of lipid-containing wastes are sensitive to the LCFAs derived from the lipid hydrolysis. A great reduction of methanogen population results in a decreased methane production [12, 14].

Retaining and protecting anaerobic digesting microbial cells inside a membrane bioreactor (MBR) can be a potential solution to overcome the problems of washout and inhibition. It has been reported that using the microorganisms encased in a semipermeable polyvinylidene fluoride (PVDF) membrane, the biogas production could be improved [15–17]. MBR was able to retain the cells; hence, it provides a better system for preventing cell washout in semicontinuous digestion processes at high organic loading rate [16, 18]. Furthermore, MBR has shown a protective effect on substrates containing inhibitors such as fruit-flavor compounds [19]. In searching the literature, no report on application of MBR to overcome LCFAs inhibition on biogas production has been found. Therefore, the objective of this work was to investigate the inhibitory effect of LCFAs on biogas production under thermophilic condition and the protective performance of MBR against LCFAs. Saturated (palmitic acid, C_16:0_, and stearic acid, C_18:0_) and unsaturated (oleic acid, C_18:1_) LCFAs were used as models of LCFA inhibitors.

The article "Inhibitory Effect of Long-Chain Fatty Acids on Biogas Production and the Protective Effect of Membrane Bioreactor" was published in 2016. Journal: Biomed Res Int.

## 2. Materials and Methods

### 2.1. Anaerobic Culture Preparation

An anaerobic culture with 22 g VS/L was obtained from thermophilic biogas plant at Borås Energy and Environment AB, Sweden. The culture was acclimated in an incubator at 55°C for 3 days prior to use. The acclimated sludge was homogenized and filtered through a sieve with a pore size of 1.0 mm in order to remove any remaining large particles. The sludge was thereafter centrifuged (Carl Padberg 77933 LE, Huber and Moser, Germany) at 30,000 rpm for 15 minutes and the supernatant was discarded. The suspended sludge was later used as an inoculum for cell containment in membrane sachets, or as free cells.

### 2.2. Synthetic Medium, Membrane, and Inhibitors

The synthetic medium was prepared as previously described [19]. It contained D-glucose, yeast extract, and nutrient broth with a concentration of 20 g/L in distilled water. The nutrient broth contained 1 g/L D(+)-glucose, 15 g/L peptone, 6 g/L sodium chloride, and 3 g/L yeast extract. The solution was homogenized and filtered using 0.2 *μ*m membrane filters. Flat plain PVDF (polyvinylidene fluoride, Durapore®) membranes were obtained from Thermo Fisher Scientific Inc. (Sweden) and used for cell encasement. PVDF membranes have a hydrophilic surface, with pore size and thickness of 0.1 *μ*m and 125 *μ*m, respectively.

Palmitic, stearic, and oleic acid were used as model LCFA inhibitors and were purchased from Sigma Aldrich (Sweden). These inhibitors were first dissolved in 2.5 mL methanol (reagent grade) in order to obtain a homogeneous solution in the reactors; thereafter, they were added to the reactors at concentrations of 0, 1.5, 3.0, and 4.5 g/L.

### 2.3. Membrane Sachet Preparation and Cell Containment Procedure

A cell containment technique was conducted following the method described in a previous study [16]. In this work, the cells were encased inside the membrane, which according to Mahboubi et al. [20] is referred to as reverse membrane bioreactor. The PVDF membranes were cut into rectangular shapes 6 × 6 cm and folded to create membrane pockets of 3 × 6 cm. The pockets were heat-sealed (HPL 450 AS, Hawo, Germany) on two sides with heating and cooling times of 4.0 and 3.5 s, leaving one side open for insertion of the inoculums. Three grams of solid inoculums was injected into the synthetic membrane pockets. The remaining open side of the sachet was sealed and the inoculum inside was carefully spread out. The inoculum containing sachets were immediately used for biogas production.

### 2.4. Anaerobic Batch Digestion Process Setup

The experiments were carried out in thermophilic batch digestion. The LCFAs were added to the reactor at concentrations of 1.5, 3, and 4.5 g/L. Reactor without addition of inhibitors was used as controls. The reactors of the free cells were performed in parallel, with otherwise identical conditions to compare the performance of membrane bioreactor in the presence of inhibitor. The experiment was conducted using 100 mL serum glass bottles with total working volume of 43.5 mL. Each reactor contained 1 mL of synthetic medium, 3 g of free cell or encased cell, 40 mL distilled water, and 2.5 mL of inhibitor solution or 2.5 mL of methanol for the control. The reactors were sealed and flushed with 80% N_2_ and 20% CO_2_ gas mix to obtain anaerobic conditions. During the biogas production process, the digesters were shaken twice a day.

The article "Inhibitory Effect of Long-Chain Fatty Acids on Biogas Production and the Protective Effect of Membrane Bioreactor" was published in 2016. Journal: Biomed Res Int.

### 2.5. Analytical Methods

Methane production was measured by Varian 450 gas chromatograph with a capillary column equipped with a thermal conductivity detector (TCD). N_2_ was used as a carrier gas, and the instrument was operated with injector and oven temperature at 75°C and 50°C, nitrogen column flow 2.0 mL/min and detector temperature at 250°C. A 0.25 mL pressure lock syringe (VICI, USA) was used for the gas sampling.

Methane production was determined as previously described by Hansen et al., 2004 [21]. The measurement of methane production was based on gas composition, releasing the gas from the reactor, changing the reactor pressure to normal pressure, and another GC measurement at this normal pressure of the reactor. The syringe used for gas sampling has a valve and, therefore, the gas inside the syringe has the same pressure as the reactor vessel in both of the measurements. The methane production was calculated from the difference of peak sizes between two measurements.

The percentage of inhibition from each treatment was used as an indicator of the inhibitory effects caused by the LCFA and calculated according to the following equation:

(1) $$\begin{array}{c} Inhibition\;\;\left(\;\%\;\right)=\frac{\left(x-y\right)}{x}\times 100, \end{array}$$

where *x* is methane production from control reactor and *y* is methane production from samples.

Volatile fatty acids (VFAs) were analyzed using a Waters® High Performance Liquid Chromatography (HPLC) system with a BIORAD Aminex® HPX-87H, 300 mm × 7.8 mm column, and 5 mM of sulphuric acid as mobile phase. It was operated at 0.6 mL/min isocratic mobile phase flow; the column temperature was set at 50°C and the VFAs were detected using a UV detector at a wavelength of 210 nm. The experiment was performed in triplicate, and the results were presented in average.

## 3. Results and Discussion

### 3.1. Inhibitory Effects of LCFAs on Biogas Production

Palmitic and stearic acids are the principal saturated LCFAs to be accumulated in anaerobic digestion process. They are known to be degraded five times slower than unsaturated acids [22]. Oleic acid is one of the most common LCFAs [23] and has the highest toxicity level among the various kinds of LCFAs, with a minimum inhibitory concentration (MIC) of 50–75 mg/L under mesophilic conditions [24–27]. However, inhibitory effects of the aforementioned LCFAs have not yet been examined under thermophilic anaerobic digestion. In this experiment, the possible inhibition effects of palmitic, stearic, and oleic acid were investigated at three different concentrations, that is, 1.5, 3, and 4.5 g/L in batch thermophilic anaerobic digestion. Reactor without addition of LCFAs was used as control. The cumulative methane productions of control as well as reactor with addition of palmitic, stearic, and oleic acid at three different concentrations are shown in Figures 1(a)–1(c), respectively.

The article "Inhibitory Effect of Long-Chain Fatty Acids on Biogas Production and the Protective Effect of Membrane Bioreactor" was published in 2016. Journal: Biomed Res Int.

Figure 1(a) shows that the methane production increased sharply in all the reactors during the first 6 days of incubation. After six days, the methane production continued at a lower rate. This indicates that the more biodegradable material was consumed within the first 6 days. The methane production started to decrease on day 4 with addition of 3 and 4.5 g/L of palmitic acid and on day 8 with addition of 1.5 g/L palmitic acid. At the end of digestion, the accumulation of methane yield with addition of palmitic acid at 0, 1.5, 3, and 4.5 g/L was 1.4, 1.1, 0.6, and 0.6 Nm^3^/kg VS, respectively. The methane production decreased by 21, 57, and 57% compared to control with addition of 1.5, 3, and 4.5 g/L. The specific methanogenic activities of control as well as reactors with addition of 1.5, 3, and 4.5 g/L palmitic acid were 0.115, 0.100, 0.055, and 0.061 Nm^3^ CH_4_/kg VS/d, respectively. A shorter time required to affect the methane production that resulted in lower cumulative methane productions at all the concentration tested compared to that of control confirmed that palmitic acid has an inhibitory effect on the thermophilic anaerobic digestion process. It has been reported that the addition of palmitic acid at a concentration of >1.1 g/L inhibited the performance of anaerobic digestion by about 50% under mesophilic conditions [28]. The result of this work shows that under thermophilic condition, methane reduction exceeding 50% was obtained when palmitic acid was added at concentration of 3 g/L. Furthermore, the maximum methane reduction was obtained with the addition of 3 g/L of palmitic acid as increasing concentration of palmitic acid up to 4.5 g/L had a similar effect with that of 3 g/L.

The article "Inhibitory Effect of Long-Chain Fatty Acids on Biogas Production and the Protective Effect of Membrane Bioreactor" was published in 2016. Journal: Biomed Res Int.

Effect of stearic acid on methane production is presented in Figure 1(b). Initially, methane was produced in all of the reactors showing that the microorganisms were able to perform at all concentrations of stearic acid added. The cumulative methane productions of reactors with addition of all tested concentrations were similar to that of control until day 4. Subsequently, the methane was produced in a lower rate compared to that of control until the end of digestion. On the last day of the digestion, the accumulated methane yield from control and the media containing stearic acid at 1.5, 3.0, and 4.5 g/L were 3.4, 1.5, 1.2, and 0.9 m^3^/kg VS, respectively. The accumulated methane yields from the media containing LCFAs correspond to 56, 65, and 74% of methane reduction with respect to control. Addition of stearic acid to the reactor also decreased the specific methanogenic activity of the reactor. The specific methanogenic activities of control were 0.181, whereas for reactors with addition of 1.5, 3, and 4.5 g/L stearic acid the specific methanogenic activities were 0.121, 0.089, and 0.078 Nm^3^ CH_4_/kg VS/d, respectively. The result shows that higher concentration of stearic acid resulted in lower methane production, which indicates an inhibitory activity of stearic acid towards anaerobic digesting microorganism. In this work, stearic acid at concentration of 1.5% is enough to reduce 50% of methane production under thermophilic condition. This is in accordance with a previous finding stating that stearic acid at a concentration of 1.5 g/L could inhibit 50 percent of the anaerobic performance under mesophilic conditions [28].

Meanwhile, the results of the effect of oleic acid study are presented in Figure 1(c). Addition of oleic acid at all tested concentration did not affect methane production until day 6 as the level of methane production was the same with that of control. Similar to those of palmitic and stearic acid, addition of oleic acid at all tested concentrations to the anaerobic digesters resulted in a lower specific methanogenic activity and a lower accumulated methane yield compared to that of control. The specific methanogenic activities of control as well as reactors with addition of 1.5, 3, and 4.5 g/L oleic acid were 0.341, 0.165, 0.067, and 0.079 Nm^3^ CH_4_/kg VS/d, respectively. The accumulated methane yields produced in the reactor with addition of oleic acid at concentrations of 0, 1.5, 3.0, and 4.5 g/L were 6.7, 3.5, 1.8, and 2.0 m^3^/kg VS, respectively. The result shows that addition of oleic acid at concentration of 1.5 g/L caused 48% reduction of methane under thermophilic condition. This concentration is higher compared to that of previous work that reported oleic acid at a concentration of 0.05–0.07 g/L could inhibit the digestion performance by about 50 percent under mesophilic conditions [26]. Oleic acid at 3 g/L exhibited strong inhibitory activity as shown by 73% methane reduction compared to that of control.

The article "Inhibitory Effect of Long-Chain Fatty Acids on Biogas Production and the Protective Effect of Membrane Bioreactor" was published in 2016. Journal: Biomed Res Int.

The results from the current work show that all the tested LCFAs reduced methane production by 50% at concentration of 1.5–3 g/L. Sousa et al. [13] reported that oleic acid had more severe effects on the methanogens than the saturated LCFAs. Furthermore, Shin et al., 2003, [24] reported that unsaturated oleic acid was more inhibitory than the saturated stearate and palmitate on the acetate degradation. The inhibitory effects of major long-chain fatty acids (LCFAs), which have 16 or 18 carbons, did not only have an effect on the acetate degradation, but also on the propionate degradation and *β*-oxidation. The adsorption of LCFAs onto the microbial cell wall or the membrane that causes damage in the microorganism's transport and protective functions is suggested to be the mechanism underlying the inhibition effect of LCFAs.

### 3.2. Performance of the Membrane Bioreactor (MBR) with Encased Cells in the Presence of Inhibitory LCFAs for Biogas Production

The MBR has been intensively studied in both batch and continuous digestion processes in order to improve the process efficiency and biogas productivity under harsh anaerobic process conditions [15–18]. The previous section showed inhibition of LCFAs on methane production under thermophilic digestion. In this work, the encased cells in the MBR system were studied in batch digestion processes, in order to investigate the potential application of this system in overcoming the inhibitory effects of LCFAs. Experiment with MBR without addition of LCFAs was used as control. Furthermore, to evaluate the performance of MBR, a conventional reactor containing free cells which run under identical condition was used as comparison. Percentage of inhibition, the accumulation of VFAs and pH were used as parameters indicating the performance of the system.

#### 3.2.1. Percentage of Inhibition

The accumulated methane yield of MBR with addition of palmitic acid is presented in Figure 2(a). As can be seen, accumulated methane yields of reactor with addition of 1.5 and 3 g/L were similar to that of control which indicates addition of palmitic acid at concentration up to 3 g/L did not affect the methane production in MBR system. However, higher concentration of palmitic acid at 4.5 g/L resulted in lower accumulated methane yield compared to that of control. The specific methanogenic activities of MBR with addition of palmitic acid were in the range of 0.032–0.049 Nm^3^ CH_4_/kg VS/h. The percentage of inhibition in the MBR with encased cells was 1.4, 5.0, and 42.3% at palmitic acid concentrations of 1.5, 3.0, and 4.5 g/L, respectively, whereas the percentage of inhibition in the reactors with free cells containing palmitic acid at concentrations of 1.5, 3.0, and 4.5 g/L was 26.1%, 70.2%, and 73.9%, respectively (Figure 3(a)). The results show that percentages of inhibition in all tested concentrations of MBR were lower than that of free cells. And this explains that MBR system was significantly less affected by the presence of palmitic acid compared to the conventional system with free cells. In addition, the inhibitory concentration (IC_50_) that reduces 50% of methane production was obtained at less than 3 g/L in free cells whereas the IC_50_ of MBR was higher than 4.5 g/L.

The article "Inhibitory Effect of Long-Chain Fatty Acids on Biogas Production and the Protective Effect of Membrane Bioreactor" was published in 2016. Journal: Biomed Res Int.

The accumulated methane yield of MBR with addition of different concentration of stearic acid is shown in Figure 2(b). The accumulated methane yield in the MBR containing stearic acid of 1.5 g/L was not significantly different with that of control. This showed that MBR could tolerate stearic acid with a concentration of 1.5 g/L, while free cells failed under the same condition (Figure 1(b)). The specific methanogenic activities of MBR with addition of stearic acid were in the range of 0.069–0.098 Nm^3^ CH_4_/kg VS/h. Furthermore, the percentage of inhibition in the bioreactor with addition of stearic acid at 1.5, 3.0, and 4.5 g/L was 54.8, 63.6, and 69.0%, respectively, for free cells and 9.1, 30.0, and 38.2%, respectively, for MBR (Figure 3(b)). The results show that IC_50_ of MBR system (>4.5 g/L) was approximately three times higher than that of free cells (<1.5 g/L).

Similar to palmitic and stearic acids, the accumulated methane yield in the MBR system with addition of oleic acid at concentration of 1.5 g/L was not significantly different with that of control (Figure 2(c)). In comparison with free cells, addition of oleic acid at the same concentration already caused 48% methane reduction. Addition of oleic acid at concentration higher than 3 g/L decreased the methane production by 33.3%. The specific methanogenic activities of MBR with addition of oleic acid were in the range of 0.065–0.090 Nm^3^ CH_4_/kg VS/h. When the performance of MBR was presented in the percentage of inhibition, the results showed that the percentage of inhibition in MBR containing oleic acid was less than 50% at all concentrations of the oleic acid. The free microbial cells in the conventional system were more severely affected by the oleic acid already at a concentration of 1.5 g/L. The inhibition was more than 50% when oleic acid concentration was increased to 3.0 and 4.5 g/L (Figure 3(c)). Hence the IC_50_ of MBR was higher than 4.5 g/L, whereas the IC_50_ of free cells was less than 1.5 g/L.

The article "Inhibitory Effect of Long-Chain Fatty Acids on Biogas Production and the Protective Effect of Membrane Bioreactor" was published in 2016. Journal: Biomed Res Int.

In general, the specific methanogenic activities of free cells were higher than that of MBR. This is most likely due to the extra resistance to the mass transfer of the substrate through the membrane. However, it did not reduce the accumulated methane yield as higher accumulated methane yield was obtained from MBR.

The results of the current work emphasize the benefit of encased cells in MBR over free cells system. In MBR system, the cells were encased in a hydrophilic PVDF membrane which theoretically is impermeable to hydrophobic compound such as LCFA. Besides, encasement increases the cell density inside the membrane which might enhance cell tolerance against the inhibitor. In addition, MBR system offers an advantage in having easier cell recovery from the bioreactor in the downstream processing unit [29].

#### 3.2.2. Volatile Fatty Acid and pH

In an anaerobic treatment, lipids are first hydrolyzed to glycerol and free LCFAs by the acidogenic bacteria. Glycerol is further converted into acetate by acidogenesis, while the LCFAs are converted into hydrogen, acetate, and/or propionate through the *β*-oxidation pathway (syntrophic acetogenesis) [30]. During the last stage of methanogenesis, the products of the previous stage are further degraded to principally carbon dioxide and methane. Under ideal operating conditions, the acid production and gas production are in balance, with the volatile acids being broken down as quickly as they are produced [31]. Thus, VFAs and pH have been widely used as fast indicators of unstable anaerobic digestion processes. Therefore, in this work, VFAs and pH were analyzed in order to investigate the performance of the encased cells in MBR system in comparison to free cells.

Tables 1 and 2 show total VFA concentrations and pH on the last day of digestion in both free cells and MBR system. The total VFA concentration and the pH in both systems were not different from the control for both free cells and MBR with addition of palmitic acid at all tested concentrations. The VFA concentrations in MBR systems with encased cells were in the range of 2.4–2.8 g/L, while the reactors with free cells were in the range of 2.1–3.2 g/L.

In the case of stearic acid, addition of LCFA at concentration higher than 3 g/L increased VFA for both free cells and MBR. The increase of VFA was followed with the decrease of pH as can be seen in Table 2. However, VFAs in free cells at addition of 4.5 g/L were two times higher than that of control, whereas under the same condition, only 25% increase of VFA was observed in MBR system. It has been reported that accumulation of VFAs above 4 g/L in the digester leads to an imbalance of anaerobic digestion process [10, 12]. In this experiment, with the addition of stearic acid at concentrations of 3.0 and 4.5 g/L the reactor with free cells resulted in an accumulation of VFA compounds to 4.4 and 5.4 g/L, respectively. In the MBR reactor, on the other hand, the VFA concentrations of 2.6 and 2.4 g/L were measured at the same concentrations of stearic acid added. In both systems with the stearic acid, the pH decreased during the incubation period (Table 2), following the concentration of VFAs (Table 1). Higher pH values were found in MBR system compared to the free cell system. The addition of stearic acid at different concentrations to the bioreactor with the free cell led to decrease in the pH from 5.97 in the control to 4.81 in the reactors with addition of 4.5 g/L stearic acid. The pH in the reactors with the encased cells, however, decreased only from 6.23 in the control to 5.79 in the reactor with the highest concentration of stearic acid.

The article "Inhibitory Effect of Long-Chain Fatty Acids on Biogas Production and the Protective Effect of Membrane Bioreactor" was published in 2016. Journal: Biomed Res Int.

Similar to stearic acid, increasing the concentration of the oleic acid added to both the systems led to an increase in the total VFA concentration. As for the other LCFAs investigated, and probably for the same reasons, the VFA accumulation was higher in the conventional system with free cells compared to MBR system with encased cells. The VFA concentrations of free cells were higher than 4 g/L in all tested concentrations. In contrast, VFA concentrations higher than 4 g/L in the MBR reactors were observed only in the reactors containing oleic acid at concentrations of 3.0 and 4.5 g/L. However, the pH values measured at the end of the incubations in both systems were not different. These results prove that MBR system with encased cells was superior to the conventional system with free cells as it shows lower percentage of inhibition, lower VFA production, and stabil pH in the presence of all tested LCFA.

In this study, the microbial cells encased in the PVDF membranes displayed less inhibition with palmitic, stearic, and oleic acid compared to the free cells. In the conventional system, the free microbial cells probably had a more direct contact with the inhibitors leading to an adsorption of the inhibitors onto the cell membrane. Gerardi [12] reported that the cell walls of methanogens lacking protective envelopes resulted in inhibitor sensitive cells. This can cause damage to the cells and lead to an unstable digestion process with a low biogas production [7]. At the end of the digestion, the higher VFA concentration in the reactor with the free cells can also be due to the fast degradation by the free cells, being readily exposed to the substrates, including the LCFAs. This resulted in high VFA concentrations in the end, since the more sensitive methanogens could not convert the VFAs as fast as they were produced by the less sensitive acid-forming bacteria. High VFA concentrations in the reactors can inhibit the activity of the methane-forming microorganisms leading to unstable digestion processes [5, 10, 24].

The article "Inhibitory Effect of Long-Chain Fatty Acids on Biogas Production and the Protective Effect of Membrane Bioreactor" was published in 2016. Journal: Biomed Res Int.

The encased cells in MBR, on the other hand, were protected by a polymeric membrane enclosing the microorganisms. The membrane could likely limit the diffusion of the inhibitors to the cells. Thereby, the microorganisms had a longer time to detoxify the medium by utilizing the LCFAs and VFAs for biogas production and maintaining them at a low concentration close to the cells. At the end of digestion, the lower VFAs concentration allowed the encased cells to perform efficiently without any negative effect from the high concentrations of VFAs; thus, a stable digestion process could be maintained. In addition, method of retaining microbial cells in the membranes provides a high cell density, meaning that the cells-to-LCFA ratio is high, thus, enabling a better acclimatization and detoxification. Alves et al. [25, 32] studied an anaerobic fixed-bed reactor that was used to prevent cells washout. It was shown that retention of cells improved the tolerance of the system in the presence of high concentrations of LCFAs in the wastewater.

It is also possible that the inhibitors could not pass through the cell pellet inside the pouches of the MBR easily, meaning that only a portion of the cells were affected by the adsorption of the inhibitors onto the cell membrane. Protection by the outer layer of cells in a dense cell pellet has previously been reported as a reason for the higher tolerance of encapsulated and flocculating yeast cells to convertible inhibitors during a second generation bioethanol production [33, 34]. Similar phenomena are likely to be present also for the encased anaerobic sludge, tightly packed in between the membrane layers.

At the same time, using membranes as cell supporting material in the MBR may lead to mass transfer limitations during the biodegradation process, especially so in static reactors only shaken once per day. This was evident from the results, with lower accumulated methane yields in the MBR compared to the reactors with free cells. MBR in continuous processes, or in batch reactors with continuous flow of the medium, would however likely display a better performance, enhancing biogas productivity in the presence of LCFAs compared to free cells, as previously observed for other inhibitory substances [15–18].

The article "Inhibitory Effect of Long-Chain Fatty Acids on Biogas Production and the Protective Effect of Membrane Bioreactor" was published in 2016. Journal: Biomed Res Int.

From the above results, it can be concluded that using PVDF membrane to enclose microbial cells in MBR reduced the inhibitory effects of palmitic, stearic, and oleic acid on the performance of microbial cells in thermophilic anaerobic degradation systems for biogas production. Thus, the degradation of lipid-containing wastes for biogas production can be run in a better balanced system as compared to the conventional system with free cells.

## 4. Conclusion

Increasing the concentration of LCFAs (palmitic, stearic, and oleic acid) to thermophilic anaerobic batch digesters led to stronger inhibitory effects on the microorganisms. Retaining cells in a membrane bioreactor (MBR) was a successful approach to decreasing the inhibitory effect of LCFAs, since a lower percentage of inhibition and more stable VFA concentration and pH value were found in MBR compared to the conventional system with free cells.

## Figures and Tables

**Figure 1:** Accumulated methane yield from reactors of free cells containing the LCFAs. (a) Palmitic acid, (b) stearic acid, and (c) oleic acid.

**Figure 2:** Accumulated methane yield from the MBR with the encased cells containing the LCFAs. (a) Palmitic acid, (b) stearic acid, and (c) oleic acid.

**Figure 3:** Percentage of inhibition in the reactors with the free cells and MBR with the encased cells in the presence of LCFAs. (a) Palmitic acid, (b) stearic acid, and (c) oleic acid.

**Table 1:** Total VFA concentration on the last day of the experiment in the reactors with the free cells and the MBR with the encased cells containing different LCFAs at different concentrations.

LCFAs	Conc. (g/L)	Total VFA concentration (g/L)	
		Free cells	Encased cells
Palmitic acid	0	2.1 ± 0.6^a^	2.4 ± 0.1^a^
	1.5	2.5 ± 0.0^a^	2.6 ± 0.0^a^
	3.0	2.6 ± 0.0^a^	2.8 ± 0.2^a^
	4.5	3.2 ± 0.0^a^	2.8 ± 0.1^a^

Stearic acid	0	2.6 ± 0.5^a^	1.8 ± 0.1^a^
	1.5	2.7 ± 0.1^a^	1.9 ± 0.0^a^
	3.0	4.4 ± 0.1^b^	2.6 ± 0.0^b^
	4.5	5.4 ± 0.2^b^	2.4 ± 0.0^b^

Oleic acid	0	4.0 ± 0.5^a^	3.4 ± 1.1^a^
	1.5	4.6 ± 0.5^a^	3.8 ± 0.1^a^
	3.0	4.5 ± 0.1^a^	4.0 ± 0.4^a^
	4.5	5.1 ± 0.2^b^	4.2 ± 1.2^b^

^a^Not significantly different from control.

^b^Significantly different from the control, *p* < 0.05, *n* = 3.

**Table 2:** pH value on the last day of the experiment in the reactors with the free cells and the MBR with the encased cells containing different LCFAs at different concentrations.

LCFAs	Conc. (g/L)	pH	
		Free cells	Encased cells
Palmitic acid	0	5.65	5.38
	1.5	5.29	5.11
	3.0	5.14	5.10
	4.5	5.18	4.90

Stearic acid	0	5.97	6.23
	1.5	5.75	6.01
	3.0	5.48	5.72
	4.5	4.81	5.79

Oleic acid	0	5.12	5.84
	1.5	5.61	5.76
	3.0	5.27	5.16
	4.5	5.25	5.20

The article "Inhibitory Effect of Long-Chain Fatty Acids on Biogas Production and the Protective Effect of Membrane Bioreactor" was published in 2016. Journal: Biomed Res Int.

## References

[1] Pavlostathis S. G., Misra G., Prytula M., Yeh D. (1996). Anaerobic processes. *Water Environment Research*.

[2] Angelidaki I., Ahring B. K. (1993). Thermophilic anaerobic digestion of livestock waste: the effect of ammonia. *Applied Microbiology and Biotechnology*.

[3] Becker P., Köster D., Popov M. N., Markossian S., Antranikian G., Märkl H. (1999). The biodegradation of olive oil and the treatment of lipid-rich wool scouring wastewater under aerobic thermophilic conditions. *Water Research*.

[4] Kim S.-H., Han S.-K., Shin H.-S. (2004). Two-phase anaerobic treatment system for fat-containing wastewater. *Journal of Chemical Technology and Biotechnology*.

[5] Quéméneur M., Marty Y. (1994). Fatty acids and sterols in domestic wastewaters. *Water Research*.

[6] Sayed S., van der Zanden J., Wijffels R., Lettinga G. (1988). Anaerobic degradation of the various fractions of slaughterhouse wastewater. *Biological Wastes*.

[7] Hanaki K., O'Nagase M., Matsuo T. (1981). Mechanism of inhibition caused by long-chain fatty acids in anaerobic digestion process. *Biotechnology and Bioengineering*.

[8] Stabnikova O., Ang S.-S., Liu X.-Y., Ivanov V., Tay J.-H., Wang J.-Y. (2005). The use of hybrid anaerobic solid-liquid (HASL) system for the treatment of lipid-containing food waste. *Journal of Chemical Technology and Biotechnology*.

[9] Wu L.-J., Kobayashi T., Li Y.-Y., Xu K.-Q. (2015). Comparison of single-stage and temperature-phased two-stage anaerobic digestion of oily food waste. *Energy Conversion and Management*.

[10] Koster I. W., Cramer A. (1987). Inhibition of methanogenesis from acetate in granular sludge by long-chain fatty acids. *Applied and Environmental Microbiology*.

[11] Rinzema A., Boone M., Van Knippenberg K., Lettinga G. (1994). Bactericidal effect of long chain fatty acids in anaerobic digestion. *Water Environment Research*.

[12] Gerardi M. H. (2003). *The Microbiology of Anaerobic Digesters*.

[13] Sousa D. Z., Salvador A. F., Ramos J. (2013). Activity and viability of methanogens in anaerobic digestion of unsaturated and saturated long-chain fatty acids. *Applied and Environmental Microbiology*.

[14] Deublein D., Steinhauser A. (2008). *Biogas from Waste and Renewable Resources*.

[15] Wikandari R., Youngsukkasem S., Millati R., Taherzadeh M. J. (2014). Performance of semi-continuous membrane bioreactor in biogas production from toxic feedstock containing d-Limonene. *Bioresource Technology*.

[16] Youngsukkasem S., Akinbomi J., Rakshit S. K., Taherzadeh M. J. (2013). Biogas production by encased bacteria in synthetic membranes: protective effects in toxic media and high loading rates. *Environmental Technology*.

The article "Inhibitory Effect of Long-Chain Fatty Acids on Biogas Production and the Protective Effect of Membrane Bioreactor" was published in 2016. Journal: Biomed Res Int.

[17] Youngsukkasem S., Chandolias K., Taherzadeh M. J. (2015). Rapid bio-methanation of syngas in a reverse membrane bioreactor: membrane encased microorganisms. *Bioresource Technology*.

[18] Youngsukkasem S., Barghi H., Rakshit S. K., Taherzadeh M. J. (2013). Rapid biogas production by compact multi-layer membrane bioreactor: efficiency of synthetic polymeric membranes. *Energies*.

[19] Wikandari R., Gudipudi S., Pandiyan I., Millati R., Taherzadeh M. J. (2013). Inhibitory effects of fruit flavors on methane production during anaerobic digestion. *Bioresource Technology*.

[20] Mahboubi A., Ylitervo P., Doyen W., De Wever H., Taherzadeh M. J. (2016). Reverse membrane bioreactor: introduction to a new technology for biofuel production. *Biotechnology Advances*.

[21] Hansen T. L., Schmidt J. E., Angelidaki I. (2004). Method for determination of methane potentials of solid organic waste. *Waste Management*.

[22] Silvestre G., Illa J., Fernández B., Bonmatí A. (2014). Thermophilic anaerobic co-digestion of sewage sludge with grease waste: effect of long chain fatty acids in the methane yield and its dewatering properties. *Applied Energy*.

[23] Lalman J. A., Bagley D. M. (2000). Anaerobic degradation and inhibitory effects of linoleic acid. *Water Research*.

[24] Shin H.-S., Kim S.-H., Lee C.-Y., Nam S.-Y. (2003). Inhibitory effects of long-chain fatty acids on VFA degradation and *β*-oxidation. *Water Science and Technology*.

[25] Alves M. M., Mota Vieira J. A., Alvares Pereira R. M., Pereira M. A., Mota M. (2001). Effects of lipids and oleic acid on biomass development in anaerobic fixed-bed reactors. Part II: oleic acid toxicity and biodegradability. *Water Research*.

[26] Hwu C.-S., Donlon B., Lettinga G. (1996). Comparative toxicity of long-chain fatty acid to anaerobic sludges from various origins. *Water Science and Technology*.

[27] Pereira A., Mota M., Alves M. (2001). Degradation of oleic acid in anaerobic filters: the effect of inoculum acclimatization and biomass recirculation. *Water Environment Research*.

[28] Pereira M. A., Pires O. C., Mota M., Alves M. M. (2005). Anaerobic biodegradation of oleic and palmitic acids: evidence of mass transfer limitations caused by long chain fatty acid accumulation onto the anaerobic sludge. *Biotechnology and Bioengineering*.

[29] Traversi D., Villa S., Lorenzi E., Degan R., Gilli G. (2012). Application of a real-time qPCR method to measure the methanogen concentration during anaerobic digestion as an indicator of biogas production capacity. *Journal of Environmental Management*.

[30] Cirne D. G., Paloumet X., Björnsson L., Alves M. M., Mattiasson B. (2007). Anaerobic digestion of lipid-rich waste-effects of lipid concentration. *Renewable Energy*.

The article "Inhibitory Effect of Long-Chain Fatty Acids on Biogas Production and the Protective Effect of Membrane Bioreactor" was published in 2016. Journal: Biomed Res Int.

[31] Weng C.-N., Jeris J. S. (1976). Biochemical mechanisms in the methane fermentation of glutamic and oleic acids. *Water Research*.

[32] Alves M. M., Vieira J. A. M., Pereira R. M. Á., Pereira M. A., Mota M. (2001). Effect of lipids and oleic acid on biomass development in anaerobic fixed-bed reactors. Part I: biofilm growth and activity. *Water Research*.

[33] Westman J. O., Bonander N., Taherzadeh M. J., Franzén C. J. (2014). Improved sugar co-utilisation by encapsulation of a recombinant *Saccharomyces cerevisiae* strain in alginate-chitosan capsules. *Biotechnology for Biofuels*.

[34] Westman J. O., Mapelli V., Taherzadeh M. J., Franzén C. J. (2014). Flocculation causes inhibitor tolerance in *Saccharomyces cerevisiae* for second-generation bioethanol production. *Applied and Environmental Microbiology*.

